# Retrospective Analysis of the Efficacy of Da Vinci Robot-Assisted Pyeloplasty in the Treatment of Ureteropelvic Junction Obstruction in Children

**DOI:** 10.1155/2021/5398858

**Published:** 2021-10-06

**Authors:** Yimeng Liu, Moudong Wu, Wei Wang, Xiong Zhan, Jinpu Peng, Nini An

**Affiliations:** Department of Pediatric Surgery, Guizhou Provincial People's Hospital, 83 Zhongshan East Road, Nanming, Guiyang, Guizhou 550002, China

## Abstract

Ureteropelvic junction obstruction (UPJO) is one of the common causes of hydronephrosis in children, and the purpose of this study was to observe the application effect of da Vinci robot-assisted laparoscopic treatment of UPJO and to investigate the safety, feasibility, and advantages of da Vinci robot-assisted laparoscopic surgery. 13 patients who underwent robot-assisted pyeloplasty (RAP) for UPJO admitted from May 2020 to March 2021 were retrospectively analyzed in our study. The clinical data among them revealed the intraoperative and postoperative indicators and complications as follows. UPJO was found on the left side in 9 patients and on the right side in 4 patients. The average operative time, blood loss, and hospital stay were 227.3 (175–310) min, 9.2 (5–30) mL, and 9.2 (6–14) days, respectively. Two cases of gross hematuria and two cases of minor urinary tract infection occurred after surgery, and the rest had no perioperative complications. The clinical treatment efficiency at postoperative follow-up was 100%. Our initial analysis showed that da Vinci robot-assisted laparoscopic surgery is a highly effective and safe option for the treatment of UPJO in children.

## 1. Introduction

Ureteropelvic junction obstruction (UPJO) is a common cause of hydronephrosis in children, and the main factors that result in UPJO include ureteropelvic junction stenosis and high ureteral orifice, ureteropelvic junction valves, external ureteral ties and adhesions, ureteropelvic polyps, junctional peristaltic dysfunction, and ectopic vessels [1–3]. The polyps occur in older children and may be present in one or all of the ureters and are prone to recurrence after surgery [4, 5]. With the popularity of prenatal ultrasonography, more and more children with hydronephrosis are being detected without clinical symptoms. For hydronephrosis caused by UPJO, the main clinical treatment is pyeloplasty. The classic surgical treatment for UPJO in children in the early years are the balloon dilatation method [6] which is introduced in 1982 and Anderson–Hynes dismembered pyeloplasty [7] which has been applied since 1995.

Schuessler et al. performed the successful laparoscopic transperitoneal pyeloplasty (C-LPP) firstly in 1993, and C-LPP has gradually replaced open surgery as the gold standard for the treatment of UPJO because of its high treatment success rate, low surgical complication rate, and low mortality rate [8, 9]. The proportion and number of laparoscopic techniques in urological surgery are increasing day by day, and their applications are becoming more widespread. As the highest level of laparoscopic system available, the da Vinci robot-assisted laparoscopic system in urological surgery is gaining more and more attention from physicians [10, 11].

In this study, 13 cases of da Vinci robot-assisted laparoscopic pyeloplasty were selected for retrospective analysis, and clinical data of patients were used to evaluate the safety as well as the effectiveness of the da Vinci robotic surgical system in the clinical management of UPJO.

## 2. Materials and Methods

### 2.1. Patient Selection

We choose 13 patients diagnosed with UPJO and underwent da Vinci robot-assisted pyeloplasty in the Guizhou Provincial People's Hospital during the period between May 2020 and March 2021. All patients signed an informed consent after the explanation about da Vinci robotic system, and this study was approved by the ethical committee of the hospital. General data of them are shown in Table 1.

### 2.2. Robotic Operative System

The da Vinci surgical system is a remote operated computer-enhanced telemanipulator for use in laparoscopic surgery and consists of two main components [12]. The control console is designed for the operated surgeon to control the movement of camera and surgical instruments. The surgical cart consisting of three robotic arms is used to maneuver a laparoscope, hold, and/or manipulate specialized surgical instruments (EndoWrist), respectively. The operating surgeon who is sitting at the console controls could receive a three-dimensional view of the surgical field while manipulating the two handles. The EndoWrist instruments have a wrist-like feature at the tip that mimics the dexterity of the human hand which can eliminate insignificant movements of the surgeon's hands through software embedded in the robot (Figure 1).

### 2.3. Surgical Procedure

The patient was placed in a 45–60° healthy-side reclined position with the lumbar region elevated after successful anesthesia, and a conventional sterilized towel was placed with an indwelling catheter (Figure 2(a)). As shown in Figures 2(b) and 2(c), an incision of approximately 1.2 cm was made at the superior border of the umbilicus (point a), then the subcutaneous layers were incised in sequence, and a pneumoperitoneum needle was inserted to create an artificial pneumoperitoneum.

The 12 mm trocar and laparoscope were inserted in sequence, and the laparoscope was placed under direct vision in the upper and lower abdomen of the affected side, respectively. Under direct vision, the skin was incised on the affected side at a point greater than 8 cm from point a (points b and d) and in the anterior superior iliac spine on the affected side at a point 8 cm from point a (point c). An 8 mm trocar was placed at points b and c, and 12 mm trocar was placed at point d. The viewing scope was placed at point a, and the da Vinci robotic arm was connected at points b and c. The laparoscopic viewing angle is 30° down at point b and c. A normal laparoscopic instrument is placed at point d to assist in the operation.

The robotic arm was operated to open the affected paracolic sulcus and the affected renal fascia and then observed the affected hydronephrosis, perinephric adhesions, and ectopic blood vessels at the pelvic-ureteral junction. The right renal pelvis and upper ureter were carefully freed, and the pelvic-ureteral junction was exposed. In case of combined ectopic vessels, the ectopic vessels can be fully released and fixed in the upper part of the renal pelvis. However, if the ectopic vessels were thin, dissection of the vessels can also be considered. The ureteral junction was incised, the excess pelvic wall was cut away, and the ureter was cut dorsally and longitudinally at the upper end. The length of the ureter was 2 to 4 cm with 6-0 absorbable wire for continuous anastomosis of the ureter and posterior wall of the renal pelvis. The F5 ureteral catheter was introduced through the d-point Trocar and inserted smoothly retrograde from the renal pelvis to the bladder. The F5 ureter was removed, and one F4.7 double J-tube was left in place, with the lower end reaching the bladder and the upper end reaching the renal pelvis. Interrupted anastomosis of the ureter and anterior pelvis and closure of the kidney with a 6-0 absorbable wire was performed (Figure 3). After checking the surgical field for any obvious active bleeding or leakage, a plasma drain tube was introduced into the trocar from point c and was placed underneath the affected pelvic anastomosis. Finally, the robotic arm and observation mirror were fully deflated after accounting all the instruments and gauze. Every trocar had to be removed and sutured and closed each incision.

### 2.4. Perioperative Indicators and Follow-Up

Intraoperative time, blood loss, intraoperative complications, postoperative hospital stay, and postoperative complications were recorded for each patient. Routine biochemical and routine blood tests were performed immediately on the 1st postoperative day. The double J stents were removed under local anesthesia and cystoscopic control depending on the patient's condition. Additionally, all patients were re-evaluated at postoperative 2 weeks, 1 month, and 3 months using renal parenchymal thickness and pelvic separation distance.

### 2.5. Statistical Analysis

Statistical significance was determined using Student's *t-*test, and data are presented as means ± SD.

## 3. Results

Mean age of a total of 13 patients was 5.0 ± 3.7 (0.17–11) years and consisted of 11 (85%) male and 2 (15%) female patients. All patients underwent preoperative confirmatory tests, including ultrasound, IUV, CT, enhanced CT, and nephogram, which showed that none of the 13 patients had any other comorbidities such as renal stones or urinary tract infections. The clinical test indicators are shown in Table 2. The mean glomerular filtration rate (GFR) of the left kidney was 43.72 ± 12.83 (21.3–64.3) mL/min, and the mean GFR of the right kidney was 39.78 ± 16.68 (8.458–55.4) mL/min; the mean percentage of GFR of the left and right kidney was 53.7% (28.4%–75.7%) and 46% (14.1%–71.4%), respectively. Mean preoperative pelvic separation was 26.2 ± 10.8 (3.1–39) mm, mean preoperative renal parenchymal thickness was 4.9 ± 3.8 (2–16) mm, and mean preoperative bed stay was 2.5 ± 2.1 (1–8) days.

All 13 patients who underwent surgery had successful surgery and recovered well after surgery, and the clinical observations are shown in Table 3. The operation time ranged from 175 to 310 min, with an average of 227.3 min; the blood loss ranged from 5 to 30 mL, with an average of 9.2 mL; the hospital stay time ranged from 6 to 14 days, with an average of 9.2 days. None of the 13 cases was operated in transit, and no intraoperative complications occurred. Two patients had postoperative carnal hematuria and two patients had minor urinary tract infection, except that, no other postoperative complications occurred.

After a 3-month follow-up, the examination of 13 patients suggested a significant reduction of postoperative upper urinary tract obstruction. Clinical data as shown in Table 4 indicated normal renal function and good recovery of bilateral renal shape. Taken together, all these data proved that the efficiency of da Vinci robot-assisted laparoscopic treatment for UPJO patients was 100%.

## 4. Discussion

Along with the development of minimally invasive surgical procedures, da Vinci robot-assisted laparoscopic surgery has been promoted for the treatment of many urological diseases, such as prostate cancer, kidney cancer, bladder cancer, pelvic-ureteral junction obstruction, and adrenal occupancy. Minimally invasive has become a trend in modern urological surgery, and robot-assisted laparoscopic techniques can improve clinical outcomes by correcting some of the deficiencies in human operating techniques, such as hand tremors and imprecise sutures [11].

UPJO is a common congenital developmental anomaly of the urinary tract. According to a survey, about 1 in 20,000 newborns has UPJO [13]. Previously, open surgery was the “gold standard” for the treatment of UPJO, with a success rate of over 90% in improving upper urinary tract obstruction [14]. Compared with conventional laparoscopic surgery, the da Vinci robot-assisted laparoscopic system has the following advantages: the field of view is three-dimensional, which is significantly better than the two-dimensional image of laparoscopy and is closer to the open surgical field of view; the system can eliminate intraoperative physiological vibrations; and the robotic control of the operating instruments can rotate flexibly in multiple directions, which enables accurate laparoscopic separation and rapid and flexible suturing. These advantages effectively reduce the difficulty of complex conventional laparoscopic surgery, reduce tissue damage, are particularly suitable for tissue and organ function reconstruction surgery, and significantly reduce the learning curve for beginners to master laparoscopic techniques [15–17].

The robot is a high-tech product that has been widely used, but there are some limitations in its application. Firstly, the high cost is hard to accept for each patient. The robot requires regular and expensive maintenance and repair every year, so patients need to pay a higher cost compared with ordinary laparoscopy, and the cost is not covered by medical insurance, so it is difficult to be applied nationwide in the short term. Secondly, because the robot has a certain volume, it occupies a larger area compared with ordinary laparoscopy and requires a separate operating room for robotic instruments. Additionally, the robotic system is lack of force feedback. Since the operator is not in direct contact with the operating lever, it cannot sense the magnitude of the operation and is prone to tissue tearing due to excessive force or suture dislodgement due to poorly knotted threads. Last but not the least, as a high-tech product, the robot has a certain rate of instrument failure and that is an issue which must be considered [18–20].

In summary, although robot-assisted laparoscopic surgery has some limitations in urological surgery where minimally invasive surgery has become a trend, it has the advantages of clear anatomical levels and delicate operation and is expected to become a new option for the treatment of UPJO in hospitals where it is available.

## 5. Conclusion

In conclusion, our data from the current study clearly suggested that the da Vinci robot-assisted laparoscopy was a safe and feasible option for the treatment of UPJO in children.

## Figures and Tables

**Figure 1:** Da vinci robotic operative system.

**Figure 2:** Trocar positions for pyeloplasty with da vinci robotic system. a, c: left-sided position; b: right-sided position. Point a: 12 mm camera trocar; point b: 8 mm trocar for da vinci endoscopic tools; point c: 8 mm trocar for da vinci endoscopic tools; point d: 12 mm trocar for conventional laparoscopic instruments.

**Figure 3:** Surgical technique of pyeloplasty with da vinci robotic system. (a) Beginning of surgery; (b) separation of pelvic ureter; (c) cutting of the renal pelvis ureter; (d) placement of the double J-tube; (e) anastomosis of the renal pelvis and ureter; (f) closure of incision.

**Table 1:** General information of patients.

Patients no.	Age (month/year)	Gender (male/female)	Body weight (kg)	Side of UPJO (left/right)	History of renal surgery (yes/no)	History of laparotomy (yes/no)
1	2 m	M	5.5	L	N	N
2	4 y	M	16	L	N	N
3	6 y	M	20	L	N	N
4	9 y	M	42	L	N	N
5	2 y	F	9	R	N	N
6	2 m	M	5	R	N	N
7	8 y	M	27	R	N	N
8	1 y	F	7.5	L	N	N
9	2 y	M	12	L	N	N
10	7 y	M	18	L	N	N
11	8 y	M	21	L	Y	Y
12	7 y	M	37	R	Y	Y
13	11 y	M	51	L	Y	N

**Table 2:** Intraoperative data of patients.

Indicators	Left kidney	Right kidney
SPECT (mL/min)	43.72 ± 12.83	39.78 ± 16.68
GFR (%)	53.72 ± 16.35	46.31 ± 16.3
Preoperative bed stay (days)	2.5 ± 2.1	
Preoperative pelvic separation	26.2 ± 10.8	
Preoperative renal parenchymal thickness (mm)	4.9 ± 3.8	

**Table 3:** Last postoperative data of patients.

Indicators	
Operative time (min)	227.3 ± 40.34
Blood loss (mL)	9.2 ± 7.0
Hospital stay time (days)	9.2 ± 2.8
Intraoperative intubation time (min)	8.5 ± 4.6
Time of drainage tube removal (days)	3.5 ± 0.8
Blood urea nitrogen value (mmol/L)	3.2 ± 1.6
Blood creatinine (*μ*mol/L)	34.7 ± 20.7
BUN/SCr	22.5 ± 9.1
eGFR (mL/min)	179.2 ± 27.7
Urinary specific gravity (SG)	1.01 ± 0.01

**Table 4:** Follow-up data of patients.

Postoperative time	Pelvic separation (mm)	Renal parenchymal thickness (mm)	Double J-tube removal time (days)
2 weeks	10.3 ± 9.9	5.0 ± 3.5	—
1 month	6.3 ± 7.0	6.0 ± 3.4	—
3 months	13.7 ± 8.3	5.8 ± 3.6	92.8 ± 16.9

## Data Availability

The simulation experiment data used to support the findings of this study are available from the corresponding author upon request.

## Abbreviations

UPJO: Ureteropelvic junction obstruction
RAP: Robot-assisted pyeloplasty
C-LPP: Laparoscopic transperitoneal pyeloplasty
GFR: Glomerular filtration rate
BUN: Blood urea nitrogen
SCr: Creatinine
SG: Urinary specific gravity.
